The article "Brain Decoding Using fMRI Images for Multiple Subjects through Deep Learning" was retracted in 2023. Reasons: unreliable results or conclusions; concerns about the data; concerns about the peer review; concerns about the citations.

# Brain Decoding Using fMRI Images for Multiple Subjects through Deep Learning

**DOI:** 10.1155/2022/1124927

**Published:** 2022-03-01

**Authors:** Muhammad Bilal Qureshi, Laraib Azad, Muhammad Shuaib Qureshi, Sheraz Aslam, Ayman Aljarbouh, Muhammad Fayaz

**Affiliations:** ^1^Department of Computer Science & IT, University of Lakki Marwat, Lakki Marwat 28420, KPK, Pakistan; ^2^Department of Computer Science, Shaheed Zulfikar Ali Bhutto Institute of Science and Technology, Islamabad 44000, Pakistan; ^3^Department of Computer Science, School of Arts and Sciences, University of Central Asia, Kyrgyzstan; ^4^Department of Electrical Engineering, Computer Engineering, and Informatics, Cyprus University of Technology, Cyprus

## Abstract

Substantial information related to human cerebral conditions can be decoded through various noninvasive evaluating techniques like fMRI. Exploration of the neuronal activity of the human brain can divulge the thoughts of a person like what the subject is perceiving, thinking, or visualizing. Furthermore, deep learning techniques can be used to decode the multifaceted patterns of the brain in response to external stimuli. Existing techniques are capable of exploring and classifying the thoughts of the human subject acquired by the fMRI imaging data. fMRI images are the volumetric imaging scans which are highly dimensional as well as require a lot of time for training when fed as an input in the deep learning network. However, the hassle for more efficient learning of highly dimensional high-level features in less training time and accurate interpretation of the brain voxels with less misclassification error is needed. In this research, we propose an improved CNN technique where features will be functionally aligned. The optimal features will be selected after dimensionality reduction. The highly dimensional feature vector will be transformed into low dimensional space for dimensionality reduction through autoadjusted weights and combination of best activation functions. Furthermore, we solve the problem of increased training time by using Swish activation function, making it denser and increasing efficiency of the model in less training time. Finally, the experimental results are evaluated and compared with other classifiers which demonstrated the supremacy of the proposed model in terms of accuracy.

## 1. Introduction

The most advanced imaging technique that is able to capture that functional part of the brain is fMRI [1]. However, task-based fMRI practices BOLD as opposed to maps of neural function in the brain. The deoxyhemoglobin concentration in the brain localizes the magnetic field. The BOLD functional magnetic resonance imaging (fMRI) shows changes to the concentration of deoxyhemoglobin arising from the regulation of a neuronal metabolism caused by activities or by spontaneity [2]. Since the activated brain regions require oxygenated blood in order to provide a significant amount of energy to neurons, the fMRI technique can distinguish both areas which are vigorous or nonvigorous in the brain underneath cognitive control. In task-based functional magnetic resonance imaging scans, the healthy participants perform various resting-state tasks during the scans [3].

The goal to practice analytical methods to classify the fMRI data is to develop efficient models that are able to predict the response of the brain stimuli in response to task-based fMRI experiments. These models imply the response of the brain with respect to the cognitive tasks performed by the human participants. The cognitive activity of the brain is involved in the construction of the brain pattern in response to the external stimulus. The purpose of this study is to accomplish the brain interpretation of the multisubject by using a predictive neural network model [4].

Various machine leaning and deep learning models have been used to analyze the fMRI data and predict the cognitive states of the brain. Various statistical models are used in machine learning to extract highly dimensional features of the brain. In deep learning, highly dimensional imaging data is converted into low dimensional subspace vector to extract features. The most commonly used deep learning-based architecture to analyze the fMRI data is convolutional neural networks [5]. The design of CNN was used from scratch with the initialization of the utilized weights from the start along with an optimizer for the effectiveness with parameters.

The goal of this study is to focus on a deep learning-based model to classify fMRI data. In the literature, various CNN methodologies have been proposed to decode brain activity. From the literature, it is observed that statistical models [6], traditional machine learning models like K-NN [7], and SVM perform well for small datasets [8] and successfully extract the region of interest, but when experiments or number of fMRI scans are increased, the amount of data received from the fMRI imaging for multisubjects becomes relatively large which results in model overfitting and increased classification errors. Even existing deep learning models like VAE [9, 10], transfer learning techniques, LSTM [11], and reconstructed fc7 layers [12] take more training time which increases computational cost. So, to overcome this, we will use a denser convolutional neural network to train high-level features. In order to train the model in less amount of time, we will be using dense connectivity CNN which will extract features with very robust learning capability, increased speed, and less training time.

We studied various types of deep learning models to classify highly dimensional-based fMRI data. To address the issue identified in the literature, we proposed an improved 3D CNN-based model to classify fMRI data which includes the combination of the best activation functions called Swish [13] along with ReLu [14] in the first few layers to convert highly dimensional data into low dimensional subspace and extract high-level features from the CNN model. The proposed method [15] first feeds raw input data into the proposed CNN model for feature extraction. At the first layer, various filters are applied to the feature maps hence reducing the feature size. Various hyperparameters were used to avoid data loss in the convolutional layers. The Swish activation function is then applied for dimensionality reduction after every layer. Later, ReLu activation function is applied before transforming the feature maps into a 1D fully connected layer. Tanh activation function is applied in every fully connected layer to minimize errors. The weights are autoadjusted. The classification is performed using a Softmax classifier.

The proposed model uses a 3D image acquired from a brain imaging experiment conducted by the Human Connectome Project (HCP) [16]. The performance of the model was examined by various performance matrixes such as F1 score, accuracy, and precision. The training time, training, and validation loss were also computed in this study to examine the model's performance. Three benchmark models were compared with the proposed model to classify the imaging data.

The rest of the paper is organized as follows.  Section 2 discusses related work.  Section 3 details the proposed improved 3D CNN architecture, and it is evaluated experimentally in Section 4. In Section 5, the produced results are discussed, and the paper is concluded in Section 6.

## 2. Related Work

The main goal of machine learning is to find the optimal parameters for its functions. Two approaches are used to make feature selection of the fMRI images. The first approach is called univariate analysis, and the second approach is called multi-voxel-based feature selection or MVPA [17]. Univariate analysis is the statistical analysis technique [18] which involves only one variable whereas multi-voxel-based pattern analysis involves multiple variables or voxels in order to identify patterns among observed conditions. We have done review of papers with MVPA-based techniques as the most recent researches are following the MVPA-based approach for feature selection whereas univariate feature selection is not preferred in the most recent researches due to its limitations on doing analysis on only one voxel.

Xu et al. [19] focused on univariate-based analysis to extract features on the voxel level and ROI level of the brain. Xu et al. used two methods to extract features to find out the better feature selection approach by using different features extracted from different human participants. The two approaches used to extract features were ANOVA followed by Kendall's coefficient. A technique called SSOMs was used in [20] for the classification of fMRI data. This technique gave better results when compared to the classic machine learning model *k*-nearest neighbor. However, as the dataset increased, SSOMs were outperformed by SVM. In order to handle highly dimensional samples, various dimensionality reduction techniques have already been applied. The very basic type of dimensionality reduction technique applied on fMRI data is called “factor models” [21]. In the existing literature, we have seen various techniques like PCA [22]; ICA [23] has been applied to the fMRI images after preprocessing. Another dimensionality reduction method called sliced inverse reduction was proposed by Tu et al. [24]. The difficulty with brain imaging is that various factors are very much correlated. Another issue is that the total number of samples is very small with very little procurement time. L1 and L2 regression [25] was used at solving the issue of high covariance across different variables by the sparse regression method. The novelty is solving the issue by sparse brain imaging retrieval technique by eliminating the noninformative region. According to Yargholi and Hossein-Zadeh [26], the key concern of decoding studies is decoding classification, but there is an inadequate consideration and much effort to improve the problem of restoring (decoding) stimulus images from fMRI records, in particular natural images. Another study [27] focused on the first contribution to a modern system of mapping connectomes based on decomposing and stitching blocks. The second contribution was to demonstrate how this structure for decomposition blocks will promote tractable link restoring with profound learning.

According to recent studies, CNN and deep learning have played an important role in the area of brain decoding. Most of the previous researches used the voxel-based classification technique and then apply the CNN model to decode the pattern [28, 29].

Preprocessing was applied to help reduce noise, SNR, head motion, and various false positive voxels which affect the accuracy score. The most frequently used classifiers for the classification of the dataset were Softmax in deep learning approaches [30] and SVM in machine learning methods. The preprocessed data for machine learning-based models was normalized using mean, cross-validation, and standard deviation whereas the deep learning-based approaches used validation and testing sets and trained the model on various epochs.

## 3. Improved 3D CNN Architecture

The 3D brain images are 3 anatomical planes as coronal, sagittal, and axial planes in the *x*, *y*, and *z* axes, respectively. The proposed model is aimed at reducing the training time with the ability to eliminate model overfitting with a reduced validation error. In the model, the fMRI data is collected from the Human Connectome Project dataset repository. The dataset is first preprocessed to remove noise caused by the human subject head movements. The HCP [31] dataset is a resting-state fMRI data where the fMRI scan is taken on healthy human subjects while the subjects are performing tasks. The spatial and temporal resolution of the HCP data is very high. The scans included the human subjects performing different tasks such as gambling, motor, language, social cognition, relational processing, working memory-related tasks, and tasks related to emotional processing. The dataset is spatially smoothed followed by temporal normalization and band pass filtering. The 3D CNN model is shown in Figure 1.

After preprocessing, the proposed convolutional neural network model is used for feature extraction. The model uses a feature map with nine different filters with stride and padding as hyperparameters to reduce feature size. The swish activation function is applied on the feature map. For dimensionality reduction, maximum pooling is applied after every convolution. To reduce training time, the dropout layer is used after every feature map followed by the batch normalization. The feature size is reduced in three feature maps followed by Swish, max pooling, and dropout layer. Finally, all feature maps are converted into a 1D fully connected layer. Deep neural networks are applied with cross-entropy to minimize the error. In the final layer, the classification model “Softmax” is applied to classify the images into correct labels. The proposed model is trained on 70% of the fMRI data. Later on, the training model is applied to validate the testing data. The classifier is evaluated in terms of accuracy, error estimation, and efficiency in the training phase. Finally, the confusion matrix is used to identify the model's classification performance and identify whether the model has correctly identified all seven classes on the fMRI HCP dataset. The comparison of Softmax is made with the SVM classifier to identify which classifier provides better accuracy. The detailed description of the proposed decoding model shown in Figure 2 is given below.

### 3.1. Input Layer

The convolutional layer stack is used in the CNN model. The multidimensional fMRI image is converted into a 2-dimensional image tensor with hyperparameters of batch size, rows, columns, and channels. To analyze the effect of initial representation over the brain decoding performance, three different input representations are fed into the deep architectures. The acquired 3D images are the slices of the brain stacked up and forming volume. During analysis, the *X* and *Y* voxels in each scan are equal to the total number of slices. The spatial dimensions of the images are in the format of 3 × 3 × 3 mm. Some of the images are rotated along with spatial dimensions. This did not involve any distortion of the image. Each slice of the brain contains a different area of the brain as the fMRI scan takes the scan of the whole brain in the form of multiple slices.

### 3.2. Convolutional Layer

The first and foremost layer in the convolutional neural network is the layer where the raw input image is placed with a series of filters. This layer is responsible for applying various filters to extract the important features. The dot product is taken of the image with filter by sliding the filter on each pixel of the image. The size of the filter with respect to the input image is considered (mxm). The final output extracted by the dot product is placed in the feature map. The feature map gives information regarding the edges, corners, and important features also called voxel extracted from the images. The feature map is then fed into other layers to extract other features.

Depth scaling given in Equation (1) is the most common technique to scale a convolutional neural network. To increase the depth of the network, more layers are added, whereas to decrease the depth of the network, the layer of convolutions is removed. The reason why depth scaling is so important is because the deeper and denser the convolutional neural network is, the most complex and richer feature the model can extract. Specially in fMRI, a more complex voxel can be extracted when the model is denser, although increasing the density of the network sometimes results in the vanishing gradient problem:

(1) $$\begin{array}{c} \text{depth}:\;d=\alpha^{\emptyset }\\ \text{s}.\text{t}.\alpha \cdot \beta^{2}\cdot \gamma^{2}\approx 2\\ \alpha \geq 1,\beta \geq 1,\gamma \geq 1. \end{array}$$

The purpose behind width scaling is to train the model efficiently. Width scaling keeps the model small resulting in reduced training time. The advantage of width scaling is that it extracts fine-grained features in less time resulting in more accuracy in less training time. It is important to note that a wider network with less density will saturate the accuracy more quickly, so width with density is used to stabilize the performance of the model in less training time. Width scaling is calculated using

(2) $$\begin{array}{c} \text{width}:\;w=\beta^{\emptyset }\\ \text{s}.\text{t}.\;\alpha \cdot \beta^{2}\cdot \gamma^{2}\approx 2\\ \alpha \geq 1,\beta \geq 1,\gamma \geq 1. \end{array}$$

### 3.3. Pooling Layer

It is a common practice to use a pooling layer right after the convolutional layer. The basic purpose of a pooling layer is to reduce the total size of the convolutional layer's feature maps which were convolved. This step is important in order to minimize the computational power. The step is performed by reducing the layer connections followed by each feature map's standalone operation. Pooling operations are of various types. It depends on the scenario regarding the pooling layer that is to be used. The two commonly used pooling operations are max pooling and average pooling. Max pooling involves the extraction of the highest element from the feature map whereas average pooling involves the extraction of the average value of the feature map where the average is extracted from all elements. The pooling layer is basically acting as a bridge which connects the two layers which are the convolutional layer and the fully connected layer. Swish activation function and ReLu will be used in the pooling layer. Swish mathematical representation is given in

(3) $$\begin{array}{c} \sigma \left(x\right)=x\frac{x}{1-e^{-x}}. \end{array}$$

### 3.4. Fully Connected Layer

The fully connected (FC) layer is comprised of neurons and weights followed by biases. This layer is used to connect the neurons between two layers. These layers of neurons are among the last few layers of the CNN model. The FC layer basically transforms the input matrix into a 1D vector. Then, it acts as an artificial neural network where the hidden layers are responsible of performing the final computation before the classification of the input images. The term flattening is used before being fed into the FC layer. The FC layer goes through more computation error calculation and weight change before starting the classification process.

### 3.5. Output Layer

The output layer is the last layer of the CNN model where classification is performed. Software activation function is mostly used to find the probability of the class which is closest to the image label.

### 3.6. Softmax Classifier

Softmax is the most commonly used activation function for the classification of the CNN model. It gives the probability of a class that is close to the image label. It is used to normalize the values between 0 and 1, and then, it gives the final output in the form of probability by dividing by their sum resulting in the output of a particular class. Softmax is only used for the output layer for classification. Softmax mathematical representation is mentioned in

(4) $$\begin{array}{c} \sigma \left(z\right)j=\frac{ezj}{\sum_{k=1}^{k}e^{z_{k}}}\text{ for}⟶j=1\cdots k. \end{array}$$

## 4. Experiments

### 4.1. Experimental Setup

For HCP [31], the setup contains experiments of different human participants ranging from under 10 to 1200 participants. The dataset used in this study contained HCP experiments with total of 45 human participants with perfect health conditions both physically and mentally. Each subject had 1-hour-long session with a 6-minute resting session in between. The position of each subject was supine. The room was dark where the experiment took place. The subject's eyes were open during the experiment. Each subject performed six different physical and cognitive tasks. The fMRI experiment type is resting-state fMRI also called rsfMRI. For this experiment, we used an Intel core i7 computer with 64 GB RAM and GeForce GTX 660 2 GB GPU. The language used to implement the model is Python using Keras 1.2.2 and TensorFlow 1.15.0. The imaging data is reshaped using Nibabel's built-in functions. The experimental setup statistics is given in Table 1.

### 4.2. Dataset Acquisition

In this study, we used the HCP dataset to understand the efficacy of the proposed model and accuracy of the classification results on the HCP dataset. The HCP dataset includes both structural MRI and rsfMRI known as resting-state fMRI images. In this study, only resting-state fMRI data is used where the participants are performing a set of tasks. rsfMRI comprises 46 healthy human participants in the scope of this study. Due to the limited computation power, the preprocessed images are of 47 human subjects collected to train our deep learning model. The fMRI images which are passed through various steps of preprocessing are thoroughly explained in the upcoming section.

In this experiment, the human participants are in a perfectly healthy condition. Each participant is exposed to different types of stimuli. In total, seven different tasks were performed by all participants. The seven different types of stimulus/tasks are named as working memory also known as WM, gambling also known as GB, motor task also known as MT, social cognition also known as SC, relational processing also known as RP, and emotional processing also known as EP. A total of about 1940 fMRI images were acquired from each human participant performing these seven types of tasks or stimuli. The fMRI data for each task was gathered in only one run. It is important to note that data from all subjects were collected performing all seven tasks. A total of more than 180000 plus images were acquired for this experimental study. The samples collected from the HCP dataset had 150000 voxels per sample. A voxel in the neuroimaging data is like a pixel in an image. In order to feed preprocessed input data, the region of interest based on voxels are already highlighted through the FSL software package in the preprocessed HCP dataset. A single voxel time series is portrayed in Figure 3.

### 4.3. Preprocessing

The acquired images were already preprocessed to remove noise and other unnecessary misalignments from the images. The first step was realignment. During the fMRI scan, it is common for the human subject to move his head. Constant head motion during the fMRI scan causes noise and sends wrong signals to the brain such that the areas of the brain get highlighted due to the increased blood flow. So, it is important to realign the images to reduce head motion. So, each fMRI 3D image is realigned to another reference image over the time of acquisition. This results in the reduced head motion effect.

### 4.4. Feature Extraction

The design of CNN was used from scratch with the initialization of the utilized weights from the start. Adam optimizer was used for the effectiveness with parameters *β*_1_ = 0.9 and *β*_2_ = 0.99. Adam optimizer [32] is a technique for gradient descent which is used for optimization in order to train deep learning models. Due to the limitations related to the memory, the size of the batch was kept 32. 0.001 learning was set as the initial learning rate. The LR was decayed by 10 every time the validation loss increased after 10 epochs. Swish activation function was used after every convolution to minimize the vanishing gradient due to backpropagation. In order to overcome the problem of overfitting data, the training of the model was stopped when the loss function was reduced to the minimum. The validation of the training set included the cross-validation approach. Five-fold cross-validation was used to validate data among the training set.

As mentioned in the previous section, the data is split into three sets [33]. The three sets are the training, validation, and testing datasets. This generalization approach will prevent the model from overfitting and also help to evaluate the model effectually. We used training data to train our CNN model, the validation set is used to choose the optimal hyperparameter, and the testing set is used to evaluate the model. The testing set (20%) is followed by the training set (70%) followed by the validation set which is 10%. Subsampling of the images was also done. The samples for all three datasets were changed for the fivefolds.

Deep learning has so many advantages; one of the most important benefits of deep learning is its reusability [34]. Traditional machine learning approaches where the features are extracted manually are outperformed by deep learning models in accuracy and efficiency. The most important advantage of this proposed CNN approach is also its reusability on similar tasks where the model is trained and tested on the validation dataset [35]. Once the model is trained in multiple epochs or iterations, the model is then tested on testing data where the images are completely different then the images where the model is trained. The transfer learning approach for the Efficient Net-based CNN model is to increase the efficiency of the model during training. The basic workflow approach is fairly similar as compared to the training time at the start. The only difference is after each convolutional layer, the activation function applied is Swish and the final output layer is left untrained.

The proposed model for brain state annotation consisted of six convolutional layers. These convolutional layers had graph filters. In total, 32 filters were used for each convolutional layer. The fully connected layers used in this model were two which were used after the flattening for the classification phase. The model takes the HCP preprocessed data in Mat format as input. The input data when fed to the convolutional neural network model propagated the information among the regions of the brain which were connected. This model generated was trained to generate graph representation followed by the classification of the labels predicted. The model is trained on 30 epochs. The batch size of the model is set to 10 subjects. The learning rate used is 0.001. The model after gaining better accuracy results is then evaluated on the testing dataset separately. After achieving high accuracy on the training model and validating through the validation dataset, the model is then evaluated on the testing dataset. L2 regularization with dropout is also used to decrease the training time. The L2 regularization value used is 0.0005, and the rate of dropout which is 0.5 was applied on all layers. The model is trained for 1000 participants. The motor task and memory task were done on diverse time windows. The fMRI volumes were 5 which were taken as input. The motor task had 10 windows whereas the memory task had 20 windows. The wrapping method was applied for task events. The layers were fine-tuned from random initialization.

### 4.5. Classification

The initial layers of CNN were responsible for feature extraction. In the next phase, the extracted features are flattened to the one-dimensional matrix. The parameters of the 1D matrix are reduced through dense hidden layers. The layer of CNN is used to classify the multiclass classification on the fMRI data. The activation function “Softmax” was used as a classifier. Softmax gave the classification score of every single fMRI image in the form of probability.

### 4.6. Evaluation

In this phase, firstly, the models built by 70% training data perform classification of the remaining 30% testing fMRI instances. Secondly, the classification results of the testing instances are evaluated by means of evaluation measures. These performance metrics are utilized to comparatively analyze various classifiers for the proposed brain decoding model. The following subsections briefly narrate the evaluation measures of accuracy, misclassification error, precision, and F1 score. Equations (5), (6), (7), and (8) are the mathematical representations of accuracy, misclassification rate, precision, and F1 score, respectively:

(5) $$\begin{array}{c} \frac{\left(\text{TP}+\text{TN}\right)}{\text{Total}}, \end{array}$$

(6) $$\begin{array}{c} \text{Error Rate}=\frac{\left(\text{FP}+\text{FN}\right)}{\text{Total}}, \end{array}$$

(7) $$\begin{array}{c} P=\frac{\text{TP}}{\text{Predicted}}, \end{array}$$

(8) $$\begin{array}{c} \text{F}1\text{ Score}=\frac{2}{1/\text{Recall}+1/\text{Precision}}. \end{array}$$

## 5. Results and Discussion

### 5.1. Classification Results on HCP Dataset

The F1 score analysis showed the performance of the classifier across all the tasks. Each task's accuracy score is mentioned in Table 2.

The average test accuracy achieved across the cross-validation of 10-fold is 91% with a random chance of 20%.

The use of the activation function followed by the domain feature transfer provided the 7% gain. Fine-tuning the convolutional layers gave no additional improvements and no impact on training time. Direct accuracy on decoding tasks was achieved by using the base efficient net model. The accuracy of 97.5% was received when the decoding model was yielded.  Table 3 shows the summary of the HCP task run details.

This also represents the high stability of the motor tasks. Fine-tuning was able to learn the specific features, but this approach might not work well when the size of the dataset is decreased as this may cause the problem of overfitting. Some distinct patterns were seen in the WM task.

At first, the generalizability shown on the HCP participants was very low with an accuracy of 30% followed by a low chance level of 12.5%. However, high variability was seen in WM and behavior tasks. The random initialization on the decoding model gave the results of 41%. The features when transferred gave an accuracy boost of 5%. The random initialization approach was used for the feature transfer. These results showed that the WM had a strong learning representation effect. Figures 4 and 5 show WM task correlation matrices.

After the validation on the main hyperparameters with a kernel of 1∗1∗1, the model recorded the high accuracy as mentioned in the previous section. *N*_ch1_ = 3, 9, 27. The model did not converge when the *N* channel reached the value of *N*_ch_ = 1. This channel was reduced to 10 epochs. In short, the CNN model was evaluated by mainly focusing on 6 stimuli. The 10 s time window for the fMRI series was used. The average test accuracy was 88%. The chance level was slightly different around 4.7%. The confusion matrix of six cerebral realms was summarized. The precision recall for each domain other than emotion was greater than 80%. According to the confusion matrix given in Table 4, the top confusions were caused by two tasks: gambling and WM.

As mentioned in the previous section, the motor tasks followed by the language tasks were easily identified. The language tasks included story and math tasks whereas the motor tasks included movements of the right and left hands followed by tongue and right and left feet. 95% score was achieved for the language task whereas an average of 94% was achieved for motor tasks. The lowest accuracy was achieved by the relational tasks followed by the working memory task. The relational processing task achieved an 81% F1 score while the average of 83% F1 score was gained by the working memory task. Some misclassification was also observed in WM, relational, and emotion tasks. The overall summary of the F1 score on different HCP tasks is given in Table 5.

The validation and training accuracy achieved between different tasks is pictorially shown in Figure 6. The loss function and prediction accuracy for the highest accuracy tasks followed by the loss function and prediction accuracy for the lowest accuracy tasks in eight epochs are illustrated.

## 6. Conclusion

The brain decoding models like CNNs and VAEs are used for feature extraction of the brain images. This is a good approach as CNNs perform better than other existing deep learning models due to high efficiency when extracting features and then classifying the images using a classifier. CNN models give better accuracy when training the images, but this includes some major limitations. The main problem with using CNN models is the issues of vanishing gradients when back propagating the images. Similarly, large datasets often cause exploding gradient problems during model training. This issue is followed by the increased computational power as CNNs-based deep learning models are trained on GPUs. Various researchers propose the technique of training the model on CPU, but this approach has its limitations. Training the model on GPU with less computational cost is another challenge. Similarly, GPU-based models take more training time but give better accuracy results. So, various researchers proposed a model where increased density can give better accuracy and increase the performance of the model. Increasing the model's density increases the accuracy, but it also increases the training time and computation. So, the proposed CNN model was implemented where the images are trained by the combination of the best activation functions. The Swish activation function overcomes the problem of vanishing gradients. Moreover, Swish activation plays an important role in reducing the computation and training time of the model. After the extraction of the features, the images were flattened to a one-dimensional matrix where the multiple hidden layers reduced the parameters and extracted the optimal features and predicted the classification results based on the extracted features using the “Softmax” classifier. Furthermore, the reliability of the proposed method was validated using the validation dataset during training followed by the testing dataset after the model training. In addition, the best-evaluated classifier followed by the existing machine learning approach was compared with the proposed model to validate the efficiency of the model. For the HCP dataset, the proposed model gave impressive results in terms of accuracy, efficiency, and specificity. The analysis of the model was also conducted in order to demonstrate the usefulness of the brain imaging analysis and feature extraction followed by classification of the model.

## Figures and Tables

**Figure 1:** 3D CNN architecture model.

**Figure 2:** Proposed CNN decoding model.

**Figure 3:** Single voxel time series.

**Figure 4:** WM task fMRI correlation matrix.

**Figure 5:** WM task frequency correlation matrix.

**Figure 6:** Prediction accuracy per 8 epochs.

**Table 1:** Parameters and values used in experiments.

Parameter	Value
Sequence	Gradient echo EPI
Repetition time (TR)	720 ms
Time to echo (TE)	33.1 ms
Flip angle	52 deg
Field of view (FOV)	208 × 180 mm (RO × PE)
Matrix	104∗90 (RO × PE)
Slice thickness	2.0 mm; 72 slices; 2.0 mm isotropic voxels
Multiband factor	8
Echo spacing	0.58 ms
Bandwidth (BW)	2290 Hz/Px

**Table 2:** Summary of accuracy score on HCP tasks.

Task	Accuracy
Emotion	94.0 ± 1.6% (mean ± SD)
Gambling	83.7 ± 4.6% (mean ± SD)
Language	97.6 ± 1.1%(mean ± SD)
Motor	97.3 ± 1.6%(mean ± SD)
Relational	89.8 ± 3.2%(mean ± SD)
Social	96.4 ± 1.0%(mean ± SD)
WM	91.9 ± 2.3%(mean ± SD)

**Table 3:** Summary of HCP task run details per subject condition on volumetric images.

Task	Volume per each run	Minimum duration in seconds	Subjects	Total runs	Condition
Emotion	405	25	1085	2	8
Gambling	284	12	1083	2	5
Language	316	12	1051	2	2
WM	274	23	1051	2	2
Cognition	232	16	1043	2	2
RP	176	18	1047	2	2

**Table 4:** Confusion matrix on HCP tasks.

Emotion	0.029	0.017	0.011	0.003	0.026	0.012	0.002
Gambling	0.025	0.829	0.003	0.001	0.115	0.022	0.005
Language	0.003	0.007	0.977	0.001	0.004	0.005	0.002
Motor	0.009	0.009	0.010	0.956	0.007	0.005	0.004
Relational	0.007	0.047	0.011	0.001	0.912	0.010	0.012
Social	0.002	0.006	0.006	0.001	0.007	0.977	0.001
WM	0.000	0.010	0.006	0.000	0.071	0.007	0.905
	Emotion	Gambling	Language	Motor	Relational	Social	WM

**Table 5:** Summary of F1 score on HCP tasks.

Task	F1 score
WM	0.84
Social	0.91
Emotion	0.92
Motor	0.94
Language	0.96
Relational	0.81

## Data Availability

Data used in the preparation of this work were obtained from the MGH-USC Human Connectome Project (HCP) database (https://ida.loni.usc.edu).
